This article has been retracted.

# Lymphangioma: A Rare Benign Cystic Pancreatic Lesion

**DOI:** 10.7759/cureus.21056

**Published:** 2022-01-09

**Authors:** Salman M Alrasheed, Maha F Alluqmani, Sabha H Almoallem, Anmar Y Alshibely, Hattan E Alharthi, Bodour S Alkhalifah, Reem M Almutairi, Saad A Alnefaie, Rawdhan K Alnahdi, Abdullah Y Alshehri, Malak O Al Dossary, Rinad F Ergsous, Malak T Bukhamsin, Ali A Alsalam, Faisal Al-Hawaj

**Affiliations:** 1 Medicine, King Saud bin Abdulaziz University for Health Sciences, Riyadh, SAU; 2 Medicine, Ibn Sina National College For Medical Studies, Jeddah, SAU; 3 Medicine, University of Dammam, Dammam, SAU; 4 Medicine, King Saud bin Abdulaziz University for Health Sciences, Jeddah, SAU; 5 Medicine, Taif University, Taif, SAU; 6 Medicine, Umm Al-Qura University, Mecca, SAU; 7 Medicine, King Saud University, Riyadh, SAU; 8 Medicine, Princess Nourah Bint Abdul Rahman University, Riyadh, SAU; 9 Medicine, King Abdulaziz University, Jeddah, SAU; 10 Medicine, Imam Abdulrahman Bin Faisal University, Dammam, SAU

**Keywords:** lymphagnioma, pancreas, cystic lesion, case report, abdominal pain

## Abstract

Pancreatic lesions are more commonly identified nowadays with the widespread use of imaging investigations. Pancreatic lesions are heterogeneous groups of pathologies with different behavior and prognosis. It is quite difficult to differentiate these lesions because of the shared clinical manifestation and the overlapping imaging features of these lesions. We report the case of a 38-year-old woman who presented with a complaint of a 3-month history of epigastric abdominal pain radiating to her back. She reported a gradual increase in the severity of the pain. She described it as sharp in quality and was exacerbated with food intake and was alleviated by oral paracetamol. There was no history of abdominal distension, weight loss, or change in appetite. Apart from asthma, she had no other comorbid conditions or previous surgeries. She was referred to have an abdominal computed tomography scan which showed a large lesion that appears to arise from the head of the pancreas and was cystic with no soft tissue component. The radiological impression was a lymphoepithelial cyst, duplication cyst, pseudocyst from previous acute pancreatitis, lymphangioma, or intraductal papillary mucinous neoplasm. The decision for open surgical removal was decided. The patient underwent laparotomy and the cystic lesion was identified as arising from the pancreatic head. Complete resection of the mass was carried out with no complications. Histopathological examination revealed cystic lesions with the presence of lymphoid cells aggregates peripherally. The lining of the channels was positive for CD31 and was negative for CD34. Such findings conferred the diagnosis of lymphangioma. Lymphangioma is a very rare tumor of the pancreas with non-specific clinical and imaging features. Complete surgical resection of the lesion is the treatment of choice and the prognosis of the tumor is favorable if the tumor was resected completely.

## Introduction

With the widespread use of imaging modalities, pancreatic lesions have been increasingly identified. In a study involving over 1400 patients who underwent magnetic resonance images of the pancreas, the incidence of cystic pancreatic lesions was approximately 20% [1]. Cystic pancreatic lesions are heterogeneous groups of pathologies with different behavior and prognosis. It is quite difficult to differentiate these lesions because of the shared clinical manifestation and the overlapping imaging features of these lesions [2]. Cystic pancreatic lesions can be broadly classified as benign or malignant lesions. The benign cystic lesions include neoplastic lesions, retention cysts, and pseudocysts. Further, the cystic pancreatic lesions may be a finding of systemic diseases such as multiple endocrine neoplasias, von Hippel-Lindau disease, and cystic fibrosis [3]. Here, we report the case of a pancreatic lymphangioma, a rare benign pancreatic cystic lesion.

## Case presentation

A 38-year-old woman presented to the general practice clinic with a complaint of a 3-month history of abdominal pain. The pain was in the epigastric area and radiated to her back. She reported a gradual increase in the severity of the pain. At the time of presentation, she scored it as 4 out of 10 on the severity scale. The pain was not awakening her from sleep. She described it as sharp in quality and was exacerbated with food intake and was alleviated by oral paracetamol. There was no history of abdominal distension, weight loss, or change in appetite.

The patient was known to have asthma that was poorly controlled mainly due to non-adherence to her medications and non-avoidance of the triggers. She had no other comorbid conditions or any surgical history of any operation. Her routine medications included inhaled salbutamol and corticosteroid. She was a non-smoker and non-alcoholic. She worked as an interior designer. The family history was positive for celiac disease and colon cancer.

She was vitally stable with a normal pulse rate, blood pressure, temperature, and respiratory rate. Abdominal examination yielded normal findings with no localized tenderness or guarding. Bowel sounds were of normal intensity and frequency. The patient underwent some laboratory investigation that included C-reactive protein (5.2 mg/dL), erythrocyte sedimentation rate (10 mm/hour), and amylase (80 U/L), which were within the reference range (Table 1).

**Table 1:** Summary of the results of laboratory findings.

Laboratory Investigation	Unit	Result	Reference Range
Hemoglobin	g/dL	14.2	13.0–18.0
White Blood Cell	1000/mL	5.8	4.0–11.0
Platelet	1000/mL	149	140–450
Erythrocyte Sedimentation Rate	mm/hr.	10	0–20
C-Reactive Protein	mg/dL	2.5	0.3–10.0
Total Bilirubin	mg/dL	0.9	0.2–1.2
Albumin	g/dL	3.8	3.4–5.0
Alkaline Phosphatase	U/L	55	46–116
Gamma-glutamyltransferase	U/L	19	15–85
Alanine Transferase	U/L	20	14–63
Aspartate Transferase	U/L	17	15–37
Blood Urea Nitrogen	mg/dL	11	7–18
Creatinine	mg/dL	0.8	0.7–1.3
Sodium	mEq/L	140	136–145
Potassium	mEq/L	3.8	3.5–5.1
Chloride	mEq/L	104	98–107
Amylase	U/L	80	40–140

In view of the patient’s family history and her chronicity of the pain, she was referred to have an abdominal computed tomography scan. The scan was performed with intravenous contrast and image acquisition was in the portovenous phase. It showed a large lesion, measuring 14.4 x 10.5 x 6.2 cm, in the maximum dimensions. The mass appears to arise from the head of the pancreas and was cystic with no soft tissue component (Figures 1-2). The radiological impression was a lymphoepithelial cyst, duplication cyst, pseudocyst from previous acute pancreatitis, lymphangioma, or intraductal papillary mucinous neoplasm.

**Figure 1:** Axial CT image demonstrates a large cystic lesion (arrow) likely arising from the pancreatic head. CT: computed tomography

**Figure 2:** Coronal CT image shows a well-defined cystic lesion (arrow) with its pressure effect. CT: computed tomography

The patient was referred to the hepatobiliary team for further management. The decision for open surgical removal was decided. The initial surgical plan included pancreaticoduodenectomy (Whipple procedure) considering the large tumor size and its location. The patient underwent laparotomy and the cystic lesion was identified as arising from the pancreatic head. Complete resection of the mass was carried out successfully without the need to resect the pancreatic head as the initial plan. The patient had an uneventful recovery. She was discharged 7 days later.

The histopathological examination of the specimen revealed cystic lesions with the presence of lymphoid cells aggregates peripherally (Figure 3). The lining of the channels was positive for CD31 (Figure 4) but was negative for CD34. The findings were in keeping with pancreatic lymphangioma.

**Figure 3:** Histopathological image shows cystic lesions with the presence of lymphoid cells aggregates peripherally.

**Figure 4:** Immunohistochemistry image shows positivity for CD31.

## Discussion

We reported a case of pancreatic lymphangioma in a young woman presenting with chronic epigastric pain. Pancreatic lymphangioma is a benign tumor that though to originate from blockage of the pancreatic lymphatic vasculature due to congenital or acquired etiologies [4]. Such acquired etiologies include previous abdominal trauma, surgical intervention, or as a complication of radiation therapy [4, 5]. In the present case, the patient did not have any relevant history to suggest an acquired etiology of the lymphangioma.

Pancreatic lymphangioma is very rare and accounts for less than 1% of all pancreatic lesions [6-9]. Pancreatic lymphangioma has non-specific clinical manifestations due to the pressure effect on the adjacent structures. As in the present case, the patient presented with abdominal pain over 3 months. Cross-sectional studies are vital in the evaluation of such masses. The pancreatic lymphangioma typically has a well-defined thin wall and homogeneous attenuation.

While the imaging studies may suggest the diagnosis of lymphangioma, histopathological examination is required to establish a definite diagnosis. As in the present case, the lymphangioma exhibit positivity for CD34 [4, 10]. The CD31, a marker of vascular endothelium, is negative in pancreatic lymphangioma [10].

Fine-needle aspiration via the endoscopic ultrasound guidance has a role in making the diagnosis of pancreatic lesions [5]. However, in the present case, we did not proceed with further diagnostic studies as the patient was symptomatic, and complete surgical resection was warranted. The prognosis of pancreatic lymphangioma is good, but recurrence may occur if the lesion was not excised completely [5].

## Conclusions

Lymphangioma is a very rare tumor of the pancreas. As the present case highlighted, the clinical and imaging features of this tumor are non-specific. Pancreatic lymphangioma should be considered in the differential diagnosis of pancreatic cystic lesions. Complete surgical resection of the lesion is the treatment of choice and the prognosis of the tumor is favorable if the tumor was resected completely.
